# Curcumin blunts epithelial-mesenchymal transition of hepatocytes to alleviate hepatic fibrosis through regulating oxidative stress and autophagy

**DOI:** 10.1016/j.redox.2020.101600

**Published:** 2020-05-30

**Authors:** Desong Kong, Zili Zhang, Liping Chen, Weifang Huang, Feng Zhang, Ling Wang, Yu Wang, Peng Cao, Shizhong Zheng

**Affiliations:** a Chinese Medicine Modernization and Big Data Research Center, Nanjing Hospital of Chinese Medicine Affiliated to Nanjing University of Chinese Medicine, Nanjing University of Chinese Medicine, Nanjing, 210022, China; b Jiangsu Key Laboratory for Pharmacology and Safety Evaluation of Chinese Materia Medica, Nanjing University of Chinese Medicine, Nanjing, 210023, China; c Department of Pharmacology, School of Pharmacy, Nanjing University of Chinese Medicine, Nanjing, 210023, China; d Department of Pharmacology, School of Integral Medicine, Nanjing University of Chinese Medicine, Nanjing, 210023, China; e Department of Oncology, Nanjing Hospital of Chinese Medicine Affiliated to Nanjing University of Chinese Medicine, Nanjing University of Chinese Medicine, Nanjing, 210022, China; f Affiliated Hospital of Integrated Traditional Chinese and Western Medicine, Nanjing University of Chinese Medicine, Nanjing, 210028, China

**Keywords:** Autophagy, Curcumin, Epithelial-mesenchymal transition (EMT), Hepatocytes, Hepatic fibrosis, Oxidative stress

## Abstract

The massive production and activation of myofibroblasts (MFB) is key to the development of liver fibrosis. In many studies, it has been proven that hepatocytes are an important part of MFB, and can be transformed into MFB through epithelial-mesenchymal transition (EMT) during hepatic fibrogenesis. In our previous study, we confirmed that curcumin inhibited EMT procession and differentiation of hepatocytes into MFB. In addition, in previous studies, it has been shown that autophagy plays an important role in the regulation of cellular EMT procession. In the current study, we showed that curcumin inhibited TGF-β/Smad signaling transmission by activating autophagy, thereby inhibiting EMT. The mechanism of degradative polyubiquitylation of Smad2 and Smad3 is likely through inhibiting tetratricopeptide repeat domain 3 (TTC3) and by inducing ubiquitylation and proteasomal degradation of Smad ubiquitination regulatory factor 2 (SMURF2), which on account of the increase of autophagy in hepatocytes. Curcumin inhibits levels of reactive oxygen species (ROS) and oxidative stress in hepatocytes by activating PPAR-α, and regulates upstream signaling pathways of autophagy AMPK and PI3K/AKT/mTOR, leading to an increase of the autophagic flow in hepatocytes. In this study, we confirm that curcumin effectively reduced the occurrence of EMT in hepatocytes and inhibited production of the extracellular matrix (ECM) by activating autophagy, which provides a potential novel therapeutic strategy for hepatic fibrosis.

## 1 Introduction

Viral, alcoholic and non-alcoholic fatty liver disease is highly prevalent in China and around the world. Nearly 40% of patients will further develop liver fibrosis, cirrhosis, and even liver failure. Among them, liver fibrosis is a common pathological procession in the development of various chronic liver diseases. Effective prevention and treatment of liver diseases are far from ideal, which is plaguing the medical community worldwide [1]. Liver fibrosis is due to excessive extracellular matrix (ECM) production and abnormal deposition of fibrous connective tissue in the liver. Pathological characteristics of liver fibrosis include proliferation and the deposition of collagen type I and collagen type III in the portal area and hepatic lobules. Moreover, the massive production and activation of myofibroblasts (MFB) is key in the procession of liver fibrosis.

Most studies on liver fibrosis have focused on the contribution of interstitial cells such as hepatic stellate cells (HSC) to the ECM, which is believed to be the main source of MFB. However, when liver fibrosis occurs, many other types of cells, including epithelial cells, bone marrow mesenchymal stem cells, and peripheral blood cells can also be transformed into MFB, thereby aggravating the course of liver fibrosis [2]. Hepatocytes, innate epithelial cells of the liver, account for about 80% of all the cells in the liver, and perform most of the liver-related functions. It was previously believed that hepatocytes were not directly involved in the production of collagen fibers; however, in many recent studies, it has been demonstrated that hepatocytes play a vital role in the occurrence and development of liver fibrosis once transformed into fibroblasts via epithelial mesenchymal transition (EMT) [[3], [4], [5], [6]]. In our previous studies, we confirmed that hepatocytes can transform into MFB-like cells via the EMT pathway after hypoxia induction and participated in collagen formation and deposition [7].

Currently, research progress in the field of anti-fibrosis drugs is slow. Antiviral and anti-inflammatory therapies that are widely used in the clinical treatment of liver fibrosis cannot prevent the ECM deposition or promote its degradation, therefore, they cannot effectively control or eradicate liver fibrosis. For a long time, the pharmacological effects and clinical development of curcumin have been a hot spot in the pharmaceutical field both at home and abroad. In our study, we showed that curcumin can effectively inhibit activation of HSC, plays a strong anti-fibrosis effect *in vivo* and *in vitro*, and has selective protective effects on hepatocytes in various types of liver injury. Moreover, we showed that curcumin can inhibit the hypoxia-induced EMT procession and reduce ECM production, which may be due to curcumin regulating the expression of transforming growth factor-β (TGF-β) signaling pathway-related proteins [7]. However, the specific underlying mechanisms involved in the regulation and control are to be elucidated, and further in-depth studies are needed.

Autophagy is an evolutionarily conserved cellular physiological procession, which plays an important role in maintaining cell development, differentiation, survival, and homeostasis. Under normal conditions, the activity of cell autophagy is low, however, under stress conditions, including cell starvation, hypoxia, and the lack of growth factors, autophagy activity can be significantly induced, thereby leading to the degradation of intracellular contents. The degradation of related molecules can change cell status by swiftly closing or activating corresponding signal transduction pathways to ensure cell survival and activity [8,9]. In previous studies, it was confirmed that autophagy is crucial in the pathogenesis of non-alcoholic fatty liver disease, liver fibrosis, liver cancer, and other liver diseases [[10], [11], [12]]. In our previous studies on the role of autophagy in hepatic fibrosis and the intervention effect of curcumin, we showed that autophagy positively correlated with the activation and proliferation of HSC. Moreover, curcumin inhibited autophagy or interfered with the expression of autophagy-related genes, thereby preventing the loss of lipid droplets in HSC and converting activated HSC into a static type. In hepatocytes, autophagy guarantees the energy supply of hepatocytes by eliminating misfolded proteins, excessive accumulation of lipids (lipolysis) and/or damaged mitochondria (mitochondrial autophagy) to maintain the homeostasis of hepatocytes [13]. In our preliminary study, we investigated the changes of autophagic flow in hepatocytes in mice with CCL_4_-induced hepatic fibrosis, and in human hepatocytes L02 under hypoxic conditions. Our findings showed that the overall autophagic level of hepatocytes in mice with hepatic fibrosis decreased. In a hypoxic environment, the autophagic level of hepatocytes first increased, then decreased gradually with time. Recent studies have shown that autophagy and EMT can regulate each other in the procession of liver injury. Autophagy can reduce the expression of Snail protein and inhibit EMT procession. Similarly, EMT can also affect the autophagic flow in hepatocytes [14]. Therefore, we hypothesize that there is a close relation between autophagic flow in hepatocytes and EMT and MFB transformation. In this study, we investigated whether the effect of curcumin on hepatocyte EMT and hepatic fibrosis progression was related to the regulation of the level of autophagy in hepatocytes.

## 2 Materials and methods

### 2.1 Animal experiments

All animal experiments were approved by the institutional and local committee on the care and use of animals of Nanjing University of Chinese Medicine (Nanjing, China), and animals received humane care according to the National Institutes of Health guidelines. Male Sprague-Dawley rats (200–250 g) were obtained from the Shanghai Slac Laboratory Animal Co., Ltd. (Shanghai, China).

Rats were randomly divided into the following five groups: control group, model group, Curcumin group (100 mg/kg), Curcumin group (200 mg/kg), and Curcumin group (400 mg/kg). The administration route and dosage of curcumin refer to our previous studies and reports [15]. A reagent consisting of 50% olive oil CCl_4_ was intraperitoneally injected into rats in all groups, except for rats in the control group, which received pure olive oil, 1 ml/kg per rat, twice a week. The treatment groups were given corresponding drugs by gavage once every other day. Rats were fed in the same quiet environment at room temperature, and had free access to food and water. After treatment and modeling, serum indexes of liver fibrosis and liver tissue injury were determined by a semi-automatic biochemical instrument and enzyme-linked immunosorbent assay.

The levels of several liver fibrosis, EMT, and the autophagy-related index were measured in liver-specific autophagy deficient mice (Alb-Cre; ATG7^fl/fl^) and their autophagy-sufficient wild type littermates (ATG7^fl/fl^), PPARα-null (PPARα^−/−^), and wild-type control (PPARα^+/+^) mice have previously been described [14]. Curcumin (200 mg/kg) was used for the treatment of the corresponding group.

### 2.2 Cell experiments

BNL CL.2 cells (mouse embryonic hepatocytes in logarithmic growth phase) were divided into five groups: normal control group, model group, curcumin low, medium, and high dose groups (10, 20, 30 μM/L). Cells were treated with TGF-β1 (2 ng·mL^−1^). Autophagy inhibitor choroquine diphosphate salt (CQ) (5 ng·mL^−1^) was used to pretreat the cells. Curcumin was given at the same time, and related indexes were determined 24 h after treatment.

Two types of *in vitro* cell models were established by constructing interference RNA (SiRNA) of BECN1 and CTR genes to transfect BNL CL.2 cells. Cells included the autophagic gene silencing model (siBECN1, model cell 1) and the control model (siCTR, model cell 2) [14]. There were 7 groups in total: normal control group, TGF-β1 stimulation group, BECN1 siRNA group, CTR siRNA group, curcumin group, BECN1 siRNA plus Curcumin group, and CTR siRNA plus Curcumin group. Except for the normal control group, all groups were treated with TGF-β1 (2 ng·mL^−1^). Moreover, the curcumin intervention group was treated with curcumin (20 μM/L). Related indexes were determined 24 h after treatment.

### 2.3 Histopathological observation

After fixation in 10% neutral formaldehyde solution, liver tissue was routinely paraffin-embedded, then sliced into 4–5 μm sections. Pathological changes in liver tissue were observed under an optical microscope after routine Hematoxylin and Eosin (H&E) staining. The deposition of collagen fibers in liver tissue was observed after Masson staining and Sirius red staining. The ISHAK liver group was used as the international standard. A pathological diagnosis of an inflammatory response score and fibrosis staging were given to all specimens according to the international standard ISHAK liver biopsy pathological score and fibrosis staging.

### 2.4 Serological indicators

The levels of alanine aminotransfease (ALT), aspartate transaminase (AST), alkaline phosphatase (ALP), lactic dehydrogenase (LDH), hydroxyproline (HYP), hyaluronic acid (HA), procollagen III (PC III) and Collagen IV in serum of rats were determined by an automatic biochemical analyzer.

### 2.5 Immunofluorescence staining

Thin sections (5 μm) of liver tissue were dewaxed with 1% bovine serum albumin. BNL CL.2 cells were preliminary treated with related reagents. Then they were incubated with corresponding primary and fluorescence-coupled secondary antibodies for immunofluorescence staining. Nuclei were stained with DAPI. A fluorescence microscope was used to visualize sections or cells and to take images blindly in a random field of vision.

### 2.6 Optical microscope

BNL CL.2 cells were digested with 0.25% trypsin to form a single cell suspension, and cells were plated into 12-well plates (1 × 10^5^ cells per well). After the cells grown to 80% confluent, cells were divided into groups according to cell experiments intervention and photographed by a microscope to evaluate morphological changes of the cells.

### 2.7 Transmission electron microscopy

BNL CL.2 cells were digested by trypsinase and collected by low-speed centrifugation. After washing with buffer solution, 3% glutaraldehyde buffer stationary solution was added to the cell precipitation for 2 h. After washing with buffer solution, cells was fixed after adding 2% osmium tetroxide buffer stationary solution, a sample gradient dehydration with gradient ethanol, and ethanol in the sample was replaced with acetone. Then the cells was penetrated into epoxy resin and embedded systerm. Ultra-thin sections of 60 nm were prepared. The changes in autophages in the cells were observed under a transmission electron microscope.

### 2.8 Fluorescent fusion protein for the detection of autophagosomes

The plasmid pcDNA3.1-GFP-LC3 was extracted according to the instructions of the kit. The pcDNA3.1-GFP-LC3 plasmid was transfected into BNL CL.2 hepatocytes by Effectene Transfection Reagent. The transfection complex was added into DMEM containing 10% fetal bovine serum according to the instructions. After 24 h of transfection, G418 was added at a final concentration of 800 mg·L^−1^. The culture medium was replaced every 3–5 days. Untransfected BNL CL.2 hepatocytes were used as negative control. After 14 days of culture, drug-resistant clones were selected from transfected cells, while all cells in the negative control group died. Transfected cells were diluted and cloned into 96-well culture plates. After 5 days of culture, the growth pore of monoclonal cells was selected and observed under inverted fluorescence microscope. Cells that showed a green fluorescence were positive cells. When the cells in the pore proliferated to about 50% fusion degree, they were successively subcultured in 24-well plates, 6-well plates, and cell culture flasks.

### 2.9 Transcriptome RNA sequencing

BNL CL.2 cells were divided into three groups: normal control group, model group (TGF-β1, 2 ng·mL^−1^), curcumin (20 μM/L), and related indexes were determined 24 h after treatment.

After total RNA was extracted and quantified, eukaryotic mRNA was enriched by magnetic beads with Oligo (dT) connections. The extracted mRNA was randomly fragmented into short fragments by Fragmentation Buffer. Fragmented mRNA was used as a template to synthesize one strand of cDNA with Random hexamers, then Buffer, dNTPs, RNaseH, and DNA polymerase I were added to synthesize the second strand of cDNA. AMPureXP beads purified double-chain products, and repaired the sticky ends of DNA to the blunt ends by using T4 DNA polymerase and Klenow DNA polymerase. Base A and joint were added to the 3 ′ends. AMPureXP beads were selected for segments, and PCR amplification was performed to obtain the final sequencing library. Illumina Hiseq 4000 was used for sequencing after quality inspection of the library. The reading length of sequencing was 2 × 150bp (PE150). After sequencing, the results were bioinformatically analyzed.

### 2.10 Western blot analysis

After cell intervention, precooled RIPA lysate was added, then PMSF and phosphatase inhibitors were immediately added, incubated on ice for 30 min, then transferred into a centrifugal tube, centrifuged at 4 °C, 15 000 r·min^−1^ for 15 min, and supernatant was obtained as the cell lysate. The protein concentration was determined by the BCA method. Electrophoresis buffer was added, and incubated in boiling water for 10 min. Proteins (50 g per sample) were resolved on SDS-PAGE gel at 100 V and transferred to a blotting membrane for 1.5 h, using skim milk powder as a blocking agent. Then, membranes were incubated with the first antibody. Membranes were washed, and then the secondary antibody was incubated and the chemiluminescent agent ECL was used for visualization.

### 2.11 Real-time PCR analysis

Total RNA was extracted using Trizol Reagent, and the RNA content was determined by an enzyme labeling instrument. Reverse transcript mRNA into cDNA and the reverse transcription products were obtained for real-time quantitative PCR. Using GAPDH as internal reference, the specific primers used for PCR were as follows. Real-time fluorescence quantitative PCR based on a comparative cycle threshold value was used to detect the relative mRNA expression. In each internal reference, the content of mRNA in each sample was standardized by the content of GAPDH.

### 2.12 Statistical analysis

Statistical software SPSS17.0 was used for variance analysis. The data were expressed as the x ± s, and the comparison between groups was analyzed by one-way ANOVA.

## 3 Results

### 3.1 Curcumin alleviates pathological damage of hepatic fibrosis

First, a classical rat model of liver fibrosis induced by a long-term low-dose CCl_4_ was established to determine the effect of curcumin on liver injury. As expected, macroscopic examination showed that CCl_4_ treatment resulted in typical hepatic fibrosis characteristics in the model group when compared with the control group. In addition, treatment with curcumin significantly improved CCl_4_-induced fibrosis injury in a dose-dependent manner (Fig. 1A). Moreover, pathological examination including H&E, Masson, and Sirius red staining indicated that hepatic chordae were arranged in a neatly manner, and there were no signs of fibrous connective tissue proliferation, pseudolobule formation, degeneration or necrosis, inflammatory cell infiltration, and fibrous tissue proliferation in the portal area in the control group. However, in the model group, the structure of hepatic lobules was destroyed, while the arrangement of the hepatic cell cord was disordered. In addition, inflammatory cell infiltration, hepatic cell edema, many fibrous tissue proliferations, and some pseudolobules were observed. Interestingly, curcumin treatment completely restored the morphology of hepatocytes to normal levels and prevented the formation of fibrous nodules (Fig. 1A). Furthermore, serology detection showed that serum levels of ALT, AST, ALP, and LDH in the model group were significantly higher than those in the control group, whereas in the curcumin group the serum levels of these enzymes were significantly decreased, and showed protective effects on normal liver function. In addition, we also examined the levels of four key markers of liver fibrosis including HYP, HA, PC III, and Collagen IV. When compared with model group, the curcumin group significantly decreased the levels of HYP, HA, PC III, and Collagen IV in CCl_4_-induced liver fibrosis rats (Fig. 1B). Overall, these results indicated that curcumin alleviated pathological damage of hepatic fibrosis.

**Fig. 1:** **Curcumin inhibits hepatic fibrosis and epithelial-mesenchymal transition and activates autophagy in vivo.** Rats were divided into five groups: control group (no CCl_4_, untreated); model group (CCl_4_ injection, no treatment); Curcumin (100 mg/kg) and CCl_4_ treatment group; Curcumin (200 mg/kg) and CCl_4_ treatment group; Curcumin (400 mg/kg) and CCl_4_ treatment group. A: Hepatic general examination of hematoxylin-eosin (HE), Masson and Sirius red stained (200 × ). B: Levels of serum alanine aminotransfease (ALT), aspartate transaminase (AST), alkaline phosphatase (ALP), lactic dehydrogenase (LDH), hydroxyproline (HYP), hyaluronic acid (HA), procollagen III (PC III) and Collagen IV. C: Immunofluorescence analysis of α-SMA and LC3 in fibrotic liver (200 × ). D: Immunofluorescence analysis of Vimentin and LC3 in fibrotic liver (200 × ). E: Protein expression of α-SMA, Vimentin, ATG-7, Beclin-1 and MAP-LC3 (x ± s, n ≥ 3). β-Actin was used as an invariant control for equal loading. Compared with the control group ^###^*P* < *0.001*; Compared with the model group *P < 0.05, **P < 0.01, ***P < *0.001*. (For interpretation of the references to colour in this figure legend, the reader is referred to the Web version of this article.)

### 3.2 Curcumin inhibits hepatocyte EMT to alleviate hepatic fibrosis

A growing number of evidence has shown that liver fibrosis is closely related to EMT [[3], [4], [5], [6], [7]]. Therefore, we put forward the hypothesis that in our previous study, curcumin alleviated hepatic fibrosis by inhibiting hepatocyte EMT. To further test this hypothesis, we determined the impact of curcumin on EMT-related markers in hepatic tissue. Obviously, tissue immunofluorescence, Western blot analysis and real-time PCR analysis showed that curcumin treatment significantly down-regulated the expression of the EMT-related marker vimentin, and fibrogenesis-related markers α-SMA in liver tissue (Fig. 1D and E). Additional *in vitro* experiments provided consistent data and showed that curcumin abolished the TGF-β-induced increase in the expression of vimentin, α-SMA, and fibronectin expression in BNL CL.2 cells (Fig. 2A and B). Collectively, these results indicated that curcumin inhibited hepatocyte EMT to alleviate hepatic fibrosis.

**Fig. 2:** **Curcumin inhibits hepatic fibrosis and epithelial-mesenchymal transition and activates autophagy in vitro.** Cell experiments were divided into five groups: control group (no TGF, untreated); model group (TGF induction, 2 ng·mL^−1^, no treatment); Curcumin (10 μM/L) and TGF induction group; Curcumin (c) and TGF induction group; Curcumin (30 μM/L) and TGF induction group. A, B and D: Protein and mRNA expression of Vimentin, Fibronectin, α-SMA, Beclin-1 (BECN1), ATG-7, ATG-5 and LC3 were detected by Western blot and Real-time PCR analysis (x ± s, n ≥ 3). β-Actin and GAPDH was used as an invariant control for equal loading. C: Fluorescent fusion protein was used to detect autophage and autophagy formation using electron microscopy (EM). Compared with the control group ^#^*P* < *0.05,*^##^*P* < *0.01,*^###^*P* < *0.001*; Compared with the model group (TGF-β, 2 ng·mL^−1^) *P < 0.05, **P < 0.01, ***P < *0.001*.

### 3.3 The activation of autophagy is associated with curcumin-induced inhibition of hepatocyte EMT and hepatic fibrosis

In previous studies, it was suggested that the induction of autophagy can regulate hepatocyte EMT [9,14]. In our study, immunofluorescent staining was performed on curcumin-treated hepatocytes using α-SMA, vimentin, and autophagy marker LC3. Curcumin treatment remarkably increased the expression of LC3 in a dose-dependent manner in BNL CL.2 cells. Through co-localization, we found that the regulation of autophagy in hepatocytes correlated with the occurrence and development of EMT and fibrosis (Fig. 1C). Moreover, curcumin treatment can dose-dependently promote the protein expression of autophagy marker LC3, Beclin-1, and ATG7 in liver tissues and hepatocytes (Fig. 1, Fig. 2B). Next, three important methods were used to determine autophagic flux in curcumin-treated hepatocytes. First, immunofluorescence of endogenous LC3 was performed on vehicle-treated and curcumin-treated hepatocytes using the fluorescent fusion protein (GFP-LC3) test. The data showed that curcumin treatment significantly increased the expression of LC3 and the autophagic flux in hepatocytes (Fig. 2C). Secondly, typical structures of autophagy were observed by transmission electron microscopy (TEM) analysis in vehicle-treated or curcumin-treated hepatocytes. Interestingly, vehicle-treated hepatocytes displayed autophagic vesicles (3 ± 2 pieces/cell) in the cytoplasm. In contrast, treatment with curcumin resulted in a remarkable increase in autophagic vacuoles (9 ± 2 pieces/cell), representing intensified autophagy (Fig. 2C). Furthermore, Western blot analysis revealed that administration of CQ abolished the inhibition effect of curcumin to TGF-β-caused increase in the expression of α-SMA and vimentin in hepatocytes (Fig. 2D). Taken together, these data suggested that the activation of autophagy was associated with curcumin-induced inhibition of hepatocyte EMT.

### 3.4 Disruption of autophagy by BECN1 siRNA impairs curcumin-induced resistance to hepatocyte EMT

Whether the activation of autophagy by curcumin was directly involved in hepatocyte EMT *in vitro*, we used BECN1 siRNA to block autophagosome formation. Morphological evaluation revealed that BECN1 siRNA canceled out curcumin (20 μM/L), and reversed the spindle-like mesenchymal shape caused by TGF-β in BNL CL.2 cells (Fig. 3A). Moreover, TEM analysis showed that autophagic vacuoles almost disappeared in the BECN1 siRNA group (Fig. 3A). Using fluorescence microscopy, it was observed that the number of GFP-LC3-labeled autophagosomes increased significantly in the siCRT group, while the number of autophagosomes decreased in the siBECN1 group (Fig. 3B). Curcumin also did not increase the levels of autophagic flux in hepatocytes. Western blot analysis and Real-time PCR results showed that when compared with the control group and the siCRT group, the siBECN1 group significantly showed reduced expression of ATG-7, Beclin-1 (BECN1), LC3, TIMP-1, and E-cadherin (epithelioid molecular recovery marker), and increased expression of fibronectin, α-SMA, and vimentin. Furthermore, we found that after autophagy was inhibited, the effect of curcumin on the regulation of hepatocyte EMT to inhibit the process of liver fibrosis was disturbed (Fig. 3C and D). In conclusion, our findings demonstrated that disruption of autophagy by BECN1 siRNA impaired curcumin-induced resistance to hepatocyte EMT.

**Fig. 3:** **Curcumin regulates autophagy of hepatocytes and inhibits epithelial-mesenchymal transition of hepatocytes.** Activated BNL CL.2 cells were exposed to siBECN1 and siCTR respectively, then treated with curcumin for 24 h. Cell experiments were divided into 7 groups: normal control group, TGF-β1 stimulation group, BECN1 siRNA group, CTR siRNA group, curcumin group, BECN1 siRNA plus Curcumin group, CTR siRNA plus Curcumin group. A: Morphological changes of liver tissue under light microscopy (200 × ) and autophagy formation under electron microscopy (EM). B: Fluorescent fusion protein was used to detect autophages. C: Western blot analysis was used to detect EMT-related, liver fibrosis-related and autophagy-related protein (x ± s, n ≥ 3). β-Actin was used as an invariant control for equal loading. D: Real-time PCR analysis was used to detect EMT-related, liver fibrosis-related and autophagy-related mRNA (x ± s, n ≥ 3). GAPDH was used as an invariant control for equal loading. Compared with the control group ^#^*P* < *0.05*, ^##^*P* < *0.01,*^###^*P* < *0.001*; Compared with the model group (TGF-β, 2 ng·mL^−1^) *P < 0.05, **P < 0.01, ***P < *0.001;* Compared with the TGF + Cur + CTR siRNA group ^&^*P* < *0.05,*^&&^*P* < *0.01,*^&&&^*P* < *0.001*.

### 3.5 Curcumin inhibits hepatocyte EMT via blocking the TTC3/SMURF2/SMADs axis

Subsequently, two questions remain, including how curcumin affects hepatocyte autophagy and how autophagy regulates EMT. According to the results of gene thermogram, curcumin can increase the gene level of autophagy, decrease the gene level of mesenchymal cell phenotype, and impact the gene level of Smads and related pathways of hepatocytes (Fig. 4A). Accumulating evidence has suggested that tetratricopeptide repeat domain 3 (TTC3), Smad ubiquitination regulatory factor 2 (SMURF2), and the TTC3/SMURF2/SMADs axis made up of the above two play important roles in EMT [16,17]. Therefore, we investigated the molecular events of curcumin inhibiting TGF-induced EMT in hepatocytes. Combined with the gene thermogram, curcumin treatment significantly reduced the protein expression of TTC3 and Smads, and increased the protein expression of SMURF2 in hepatocytes (Fig. 4B). Moreover, real-time PCR analysis showed that mRNA levels of TTC3, SMURF2, and Smads were down-regulated in curcumin-treated hepatocytes (Fig. 4C). Furthermore, immunofluorescence analysis confirmed that autophagy could indeed affect the expression of TTC3 and Smad2/Smad3 (Fig. 4D and E). The increase in autophagy resulted in a decrease in TTC3, which further resulted in the enhancement of SMURF2 function. SMURF2 can inhibit formation of the Smad2/Smad3 complex and eventually lead to blockade of the EMT procession in hepatocytes. In conclusion, curcumin inhibited TGF-β-induced EMT through autophagy, thereby affecting the TTC3/SMURF2/SMADs axis.

**Fig. 4:** **Curcumin inhibits hepatocyte epithelial-mesenchymal transition via blocking TTC3/SMURF2/SMADs axis.** Activated BNL CL.2 was exposed to siBECN1 and siCTR respectively, and then treated with curcumin for 24 h. The resulting cells were induced with TGF-β (2 ng·mL^−1^) or interfered with curcumin (20 μM/L). A: Gene thermogram for BNL CL.2 treatment with curcumin or not, which induced by TGF-β (2 ng·mL^-1^) in advance. B–C: Western blot and Real-time PCR analysis were used to detect the expression of TTC3, SMURF2, Smad2, Smad3, α-SMA, Vimentin, Beclin-1 (BECN1) and LC3 (x ± s, n ≥ 3). β-Actin was used as an invariant control for equal loading. GAPDH was used as an invariant control for equal loading. D: Immunofluorescence detection of autophagy, Smads, TTC3-related proteins expressions. Compared with the control group ^#^*P* < *0.05*, ^##^*P* < *0.01,*^###^*P* < *0.001*; Compared with the model group (TGF-β, 2 ng·mL^−1^) *P < 0.05, **P < 0.01, ***P < *0.001*.

### 3.6 Curcumin promotes autophagy activation through regulating AMPK/PI3K/AKT/mTOR signaling

Numerous studies have demonstrated a crucial role for AMPK (Adenosine 5′-monophosphate (AMP)-activated protein kinase)/PI3K (Phosphoinositide 3-kinase)/AKT (PKB, Protein Kinase B)/mTOR (Mammalian target of rapamycin) signaling in autophagy induction [18]. We hypothesized that the regulation of AMPK/PI3K/AKT/mTOR signaling by curcumin plays a pivotal role in the induction of autophagy. To test this hypothesis, we employed different biological methods to investigate the effect of curcumin on AMPK/PI3K/AKT/mTOR signaling in hepatocytes. First, Western blot analysis indicated that curcumin treatment significantly increased the protein expression of AMPK and decreased the protein expression of mTOR in hepatocytes (Fig. 5A). Secondly, real-time PCR analysis showed that mRNA levels of AMPK were up-regulated, and that mRNA levels of mTOR were down-regulated in curcumin-treated hepatocytes (Fig. 5B). Several reports have recently provided strong evidence for the involvement of PPARα and ROS in the induction of autophagy in response to chemotherapy-induced stress [19,20]. As expected, in our study, we showed that curcumin activated peroxisome proliferators-activated receptor-α (PPAR-α) to decrease the ROS level and oxidative stress, and increase the GSH level in hepatocytes (Fig. 5A, B and 5C). Overall, these findings suggested that curcumin promoted autophagy activation through regulating PPARα and oxidative stress, to affect downstream AMPK/PI3K/AKT/mTOR signaling.

**Fig. 5:** **Curcumin promotes autophagy activation through regulating AMPK/PI3K/AKT/mTOR signaling.** Cell experiments were divided into five groups: control group (no TGF, untreated); model group (TGF induction, 2 ng·mL^−1^, no treatment); Curcumin (10 μM/L) and TGF induction group; Curcumin (c) and TGF induction group; Curcumin (30 μM/L) and TGF induction group. A–B: Western blot and Real-time PCR analysis were used to detect the expression of PPARα, AMPK, mTOR, SQSTM1, α-SMA, Vimentin and LC3 (x ± s, n ≥ 3). β-Actin was used as an invariant control for equal loading. GAPDH was used as an invariant control for equal loading. ROS、GSH was tested with the corresponding kit. Compared with the control group ^#^*P* < *0.05*, ^##^*P* < *0.01,*^###^*P* < *0.001*; Compared with the model group (TGF-β, 2 ng·mL^−1^) *P < 0.05, **P < 0.01, ***P < *0.001*.

### 3.7 PPARα upregulation and oxidative stress inhibition is required for curcumin to induce autophagy activation and inhibit hepatocyte EMT

Next, we further used PPARα inhibitor GW6471 to analyze the relationship between PPARα and the promotion of autophagy in hepatocytes. Interestingly, inhibition of PPARα impaired the activity of curcumin on AMPK, and the inhibitory effect of curcumin on PI3K/AKT/mTOR signaling and autophagy axis. Of note, the inhibition of PPARα can completely abrogate the curcumin-induced LC3-II conversion. Moreover, the inhibition of PPARα can dramatically eliminate the regulatory effects of curcumin on hepatocyte EMT and fibrinogenesis (Fig. 6A and B). Lastly, when compared with the TGF plus Curcumin group, the TGF plus Curcumin plus GW6471 group showed increased levels of ROS and oxidative stress, and decreased levels of GSH (Fig. 6C). Taken together, these data showed that PPARα upregulation was required for curcumin to induce autophagy activation and inhibit hepatocyte EMT.

**Fig. 6:** **PPARα upregulation is required for curcumin to induce autophagy activation and inhibit hepatocyte epithelial-mesenchymal transition**. PPAR-α activity of BNL CL.2 inhibited by GW6471 treatment. And cells were induced with TGF-β (2 ng·mL^−1^) or interfered with curcumin (20 μM/L). A–B: Western blot and Real-time PCR analysis were used to detect the expression of PPARα, AMPK, mTOR, SQSTM1, α-SMA, Vimentin and LC3 (x ± s, n ≥ 3). β-Actin was used as an invariant control for equal loading. GAPDH was used as an invariant control for equal loading. ROS and GSH were tested with the corresponding kit. Compared with the control group ^#^*P* < *0.05*, ^##^*P* < *0.01,*^###^*P* < *0.001*; Compared with the model group (TGF-β, 2 ng·mL^−1^) *P < 0.05, **P < *0.01*; Compared with the TGF plus curcumin group ^$^*P* < *0.05,*^$$^*P* < *0.01*.

### 3.8 Curcumin blunts hepatocyte EMT to alleviate hepatic fibrosis through regulating autophagy signaling *in vivo*

To elucidate whether curcumin blunted hepatocyte EMT to alleviate hepatic fibrosis through regulating autophagy signaling, and whether the above results depend on the activation of PPAR and inhibition of oxidative stress by curcumin *in vivo*, two classical murine liver fibrosis models induced by carbon tetrachloride were established. Fortunately, we obtained liver-specific autophagy deficient mice (Alb-Cre; ATG7^fl/fl^) and their autophagy-sufficient wild type littermates (ATG7^fl/fl^) from the Nanjing University. In addition, we also generated vitamin A-coupled liposomes carrying PPARα siRNA to knock down PPARα expression in hepatocytes (PPARα^−/−^). Using these animal models, we demonstrated that pathological changes and collagen deposition in the liver were more severe, and that curcumin could not reverse it when liver-specific autophagy was inhibited (Fig. 7A). Moreover, inhibition of liver-specific autophagy can completely abrogate the curcumin-induced LC3 conversion. Liver-specific autophagy deficiency can impair the inhibitory effect of curcumin on the TTC3/SMURF2/SMADs axis. Moreover, the inhibition of liver-specific autophagy can dramatically eliminate the regulatory effects of curcumin on hepatocyte EMT and fibrinogenesis (Fig. 7B). Furthermore, our findings showed that when compared with wild type mice, the phenomena of hepatic fibrosis were obvious in PPARα knockout mice, and the level of oxidative stress, the expression of Recombinant Nicotinamide Adenine Dinucleotide Phosphate Oxidase 1 (NOX1) increased, the effects induced by curcumin (enhanced autophagy, inhibited EMT and decreased hepatic fibrosis) were weakened (Fig. 7C and D). Overall, these results demonstrated that curcumin blunted hepatocyte EMT to alleviate hepatic fibrosis through targeting PPARα to regulate autophagy signaling *in vivo*.

**Fig. 7:** **Curcumin blunts hepatocyte epithelial-mesenchymal transition to alleviate hepatic fibrosis through regulating autophagy signaling in vivo.** ATG7^fl/fl^, Alb-Cre; ATG7^fl/fl^ mice and PPARα^+/+^, PPARα^−/−^mice were used in this study. 50% olive oil CCl_4_ reagent was intraperitoneally injected to establish an animal model of liver fibrosis in Model, ATG7^fl/fl^, Alb-Cre; ATG7^fl/fl^, PPARα^−/−^ group. The corresponding group was treated with curcumin (200 mg/kg). A and C: HE, Masson and Sirius red stained liver, and immunofluorescence analysis of liver α-SMA and LC3 (200 × ). B and D: Western blot analysis was used to detect the expression of PPAR-α, NOX1, Beclin-1, LC3, TTC3, SMURF2, Smads, α-SMA, Vimentin and ATG7 (x ± s, n ≥ 3). β-Actin was used as an invariant control for equal loading. Compared with the control group ^#^*P* < *0.05*, ^##^*P* < *0.01,*^###^*P* < *0.001*; Compared with the model group *P < 0.05, **P < 0.01, ***P < *0.001*. (For interpretation of the references to colour in this figure legend, the reader is referred to the Web version of this article.)

## 4 Discussion

EMT is a dynamic transition from the epithelial phenotype to the mesenchymal phenotype. A large number of studies have shown that EMT and its intermediate state play an important role in the invasion and metastasis of various diseases [21]. EMT has long been identified as a key role of cancer cells [22]. In the past, studies on renal and intestinal fibrosis also focused on EMT [23,24]. Most studies on liver fibrosis EMT focused on HSC cells, nevertheless, hepatocyte EMT has also been proven to be an important biological procession in liver pathophysiology. Any chronic liver injury can lead to the transformation of hepatocytes into MFB through the EMT procession, resulting in liver disease [25]. In our previous studies, we analyzed the effect of curcumin on hepatocyte EMT and its relationship with the attenuation of chronic liver injury. Our findings showed that curcumin significantly reversed the fibrosis and hepatocyte mesenchymal morphology of rats treated with CCl_4_, and significantly reduced the expression of EMT markers. However, the underlying mechanism of action remains to be elucidated.

In previous studies, it was shown that autophagy is involved in the regulation of EMT. Autophagy is a complex metabolic procession through which cells degrade dysfunctional or useless cytoplasmic components. Autophagy is a self-phagocytosis procession in most cells, and is responsible for maintaining cell homeostasis. When a cell experiences starvation or is getting rid of damaged organelles and redundant or misfolded proteins, autophagy rapidly increases [26]. In this study, we demonstrated that curcumin increased the expression of autophagic proteins in a dose-dependent manner in both the rat model and in cell experiments. To clarify the relationship between curcumin, EMT, and autophagy, two *in vitro* models were established by the siRNA approach: a normal autophagy model and a loss of autophagy model. As expected, curcumin attenuated hepatocyte EMT by enhancing autophagy.

Although we have confirmed that curcumin can inhibit the EMT procession by enhancing autophagy of hepatocytes, we still face two problems. One is how does autophagy affect EMT procession, the other is how does curcumin affect autophagy. In previous studies, it was shown that autophagy can affect the EMT procession of hepatocytes by regulating the transcription factor Snail. However, we hypothesize that autophagy in the cytoplasm may inhibit EMT procession by directly affecting signal transduction of the Smad protein. We know that Smad-dependent signal transduction is related to the EMT procession in hepatic fibrosis [27]. Sung et al. demonstrated that inhibition of Smad signaling reduced the EMT procession and the accumulation of ECM in renal fibrosis [28]. To analyze the relationship between Smad, autophagy and EMT, we established an *in vitro* model of autophagy interference. Our findings showed that TGF stimulated the expression of EMT-related proteins and increased the expression levels of p-Smad2/3 and Smad2/3. Curcumin can increase the expression of autophagic protein and reduce the transmission of Smad pathway. In addition, Smad ubiquitination regulatory factor 2 (SMURF2) is one of the E3 ubiquitination ligases, and the most critical factor in the ubiquitination procession. It can specifically identify different substrates and inhibit the TGF-beta 1/Smad signaling pathway, thereby inhibiting or delaying the procession of liver fibrosis. TTC3 is an E3 ubiquitin ligase that works as a specific terminal regulator of Akt/mTOR signal transduction. Akt/mTOR signal transduction is the core pathway of cell survival [16]. Kim et al. found that overexpression of TTC3 resulted in a decrease in the SMURF2 level, which further contributed to the TGF-induced EMT procession and differentiation of MFB [17]. In our study, we showed that curcumin decreased TTC3 expression and increased SMURF2 expression. In conclusion, all these results suggested that curcumin can influence the transmission of TTC3/SMURF2/SMADs axis through activating autophagy.

Next, we aimed to explain how curcumin affects the autophagy procession. Peroxisome proliferator-activated receptors (PPARs) are adhesive-activated nuclear receptors involved in transcriptional regulation of lipid metabolism, oxidative stress, energy balance, inflammation, and atherosclerosis [19]. Three known types of PPARs have been described: PPAR-α,PPARδ/β, and PPAR-γ. Choi et al. found that capsaicin can improve liver fibrosis by activating PPAR-γ to inhibit the TGF-β1/Smad pathway [20]. PPAR-α is mainly expressed in liver tissue and hepatocytes. By regulating the expression of fatty acid oxidation-related genes, it is crucial for hepatic adipocyte differentiation, lipid storage, lipid transport, and fatty acid oxidation. Zhao et al. found that PPAR-α agonists can reduce cholestatic liver injury induced by alpha-naphthalene isothiocyanate (ANIT) [29]. Many studies performed in our laboratory confirmed that curcumin may be a potential ligand of PPAR-γ, and inhibits the activation of HSC and the occurrence and development of liver fibrosis by activating PPAR-γ, which is highly expressed in HSC. In addition, curcumin has the potential to activate PPAR-α in hepatocytes. In this study, we showed that curcumin restored the expression of PPAR-α, the activation of which resulted in a decrease in the oxidative stress level. As a result, curcumin increased AMPK in a dose-dependent manner and decreased PI3K/AKT/mTOR expression, regulated the upstream signals of autophagy, thereby enhancing autophagy, which has been reported in several studies [18,30]. To further confirm the experimental results, we used GW6471 to inhibit the expression of PPAR-α. We showed that the indicators of liver fibrosis and EMT were increased, and that the expression of autophagy protein was decreased, which decreased the therapeutic effect of curcumin. Finally, we used PPAR-α and liver autophagy-specific knockout mice to further verify the results, which were consistent with the previous findings.

In conclusion, our findings confirm that curcumin effectively improved CCl_4_-induced hepatic fibrosis induced in rats and inhibited the EMT procession of hepatocytes. This may be due to the enhancement of autophagy level of hepatocytes by curcumin (Fig. 8). Therefore, our data provides further support for the anti-fibrosis mechanism of curcumin. Curcumin is expected to become an effective drug for the treatment of liver fibrosis and provide effective reference and guidance for clinical treatment.

**Fig. 8:** Proposed mechanisms underlying curcumin blunts hepatocyte epithelial-mesenchymal transition through regulating oxidative stress and autophagy.

## Declaration of competing interest

The authors declare no conflict of interest.
